# LncRNA PTCSC3 is upregulated in osteoporosis and negatively regulates osteoblast apoptosis

This article has been retracted.

**DOI:** 10.1186/s12920-022-01182-3

**Published:** 2022-03-16

**Authors:** Xingchao Liu, Mingliang Chen, Qinghe Liu, Gang Li, Pei Yang, Guodong Zhang

**Affiliations:** 1 Orthopedics Department, Hebei Yanda Hospital, Yanjiao Development Zone, Sanhe City, Langfang City, 065201 Hebei Province People’s Republic of China; 2 Orthopedics Department, Beijing Chao-Yang Hospital, Capital Medical University, No 8 Gongtinan Road, Beijing, 100020 People’s Republic of China

**Keywords:** Osteoporosis, lncRNA PTCSC3, Osteoblasts, Apoptosis

## Abstract

**Background:**

It is known that long non-coding RNA (lncRNA) PTCSC3 is involved in thyroid cancer and glioma, but its function in osteoporosis is unknown. The aim of our study was to investigate the role of lncRNA PTCSC3 in osteoporosis.

**Methods:**

A total of 80 patients with osteoporosis (4 clinical stages) and four corresponding groups of healthy controls were enrolled. Plasma PTCSC3 levels in the 80 osteoporosis patients and 80 healthy volunteers were measured using RT-qPCR. The diagnostic potential of plasma PTCSC3 for osteoporosis was evaluated by ROC curve analysis with healthy volunteers as the true negative cases and corresponding osteoporosis patients as the true positive cases.

**Results:**

PTCSC3 was upregulated in osteoporosis patients compared with healthy controls. PTCSC3 levels increased with osteoporosis stages increasing, but not with healthy controls aging. PTCSC3 overexpression separated each stage of osteoporosis from corresponding controls. PTCSC3 overexpression promoted while PTCSC3 silencing inhibited osteoblast apoptosis. However, PTCSC3 overexpression and silencing showed no significant effect on osteoclast apoptosis. LncRNA PTCSC3 was upregulated in osteoporosis and negatively regulated osteoblast apoptosis.

**Conclusion:**

LncRNA PTCSC3 may serve as a potential therapeutic target for osteoporosis.

**Supplementary Information:**

The online version contains supplementary material available at 10.1186/s12920-022-01182-3.

## Background

Analyses on the human transcriptome have revealed that only 1/5 of transcripts are associated with protein-coding genes, while most of the genes in the human genome transcribe long non-coding RNAs (lncRNAs) [1, 2]. Despite lacking protein-coding capacity, lncRNAs are critical determinants in regulating gene expression and participate in cell development and differentiation [3]. LncRNAs also participate in the development and progression of human diseases, and regulating lncRNAs is a promising therapeutic target for the treatment of various types of diseases [4, 5]. To date, the functions of only a small portion of lncRNAs have been characterized, and the clinical applications of lncRNAs are limited by their unclear functionality.

Osteoporosis is a common clinical bone disease, affecting more than 200 million people worldwide [6]. It is estimated that about 40% of females and 30% of males will develop osteoporosis during their lifetime [7]. Osteoporosis occurrence is closely correlated with aging [8]. With the population aging, its incidence is predicted to further increase in the near future [8]. LncRNAs are key players in osteogenic differentiation, indicating their potential involvement in osteoporosis [9, 10]. LncRNA PTCSC3 is a recently characterized tumor-suppressive lncRNA in thyroid cancer and glioma [11–13]. Our preliminary deep sequencing data analysis (Additional file 1: Fig. S1) revealed altered PTCSC3 expression in osteoporosis and its close correlation with disease stages, suggesting the involvement of PTCSC3 in osteoporosis. In the present study, we explored the functions of lncRNA PTCSC3 in osteoporosis and found that lncRNA PTCSC3 downregulation may be a potential therapeutic target for osteoporosis.

## Methods

### Subjects

A total of 80 patients with osteoporosis who were admitted to Beijing Chao-Yang Hospital, Capital Medical University from January 2016 to January 2018 were enrolled in this study. All patients were diagnosed according to the WHO criteria. The inclusion criteria were (1) osteoporosis patients with complete medical records of the past 5 years and (2) patients who were willing to participate. The exclusion criteria were (1) patients who had been treated before admission and (2) patients with other types of bone diseases. According to the staging of osteoporosis, there were 20 cases at stage I (no visible symptoms), 21 cases at stage II (detectable through bone-density tests), 15 cases at stage III (bones are thin and can be broken under stress that they normally could withstand), and 24 cases at stage IV (Increased pain and disability). Four groups of healthy controls were also enrolled to match the age and gender distribution of the corresponding osteoporosis groups (stages). All healthy controls received systemic physical examinations in the aforementioned hospital, and all indicators were within the normal range. This study was approved by the Ethics Committee of this hospital, and all patients and healthy controls signed informed consent. Table 1 lists the general information of all participants.

**Table 1:** General information of all participants

	Control I	Stage I	ControlII	Stage II	Control III	Stage III	Control IV	Stage IV
Cases	21	20	22	21	17	15	24	24
Gender								
Male	9	8	11	10	10	9	14	13
Female	12	12	11	11	7	6	10	11
Age (years)	34.3 ± 4.4	34.1 ± 4.2	41.2 ± 3.7	42.0 ± 4.6	51.6 ± 4.0	52.1 ± 3.9	60.6 ± 4.8	61.1 ± 4.7

### Plasma samples and cells

Blood (5 ml) was extracted from the elbow veins of healthy controls and patients before treatment. Blood was transferred to citrate-treated tubes and centrifuged at 1200 × *g* at 4 °C for 10 min to collect plasma samples.

Primary osteoblasts (406OA-05A, derived from an adult with osteoporosis) were purchased from Sigma-Aldrich (St. Louis, MO, USA). Osteoclasts from a stage IV osteoporosis female were isolated and cultured as previously described [14]. Briefly, bone marrow cells were isolated from bone tissues by flushing the long bones using 1 × PBS and red blood cell lysis. CD11b + monocytes were magnetically isolated using microbeads and cultured in osteoclast differentiation media. Differentiated osteoclasts were detached using Accutase, transferred to new tubes, and centrifugated at 350 g for 5 min. Cells were then collected and resuspended in ice-cold PSE. Osteoclasts with more than 3 nuclei were considered mature osteoclasts and sorted using FACS Aria IIu, collected in FBS, and cultured. Cells of passage 5–7 were harvested for subsequent experiments.

### RNA extraction and real-time quantitative PCR (RT-qPCR)

To detect PTCSC3 expression, total RNAs were extracted using RNAzol® RT RNA Isolation Reagent (Sigma-Aldrich, St. Louis, MO, USA) and reverse transcribed into cDNAs using RevertAid RT Reverse Transcription Kit (Thermo Fisher Scientific). All PCR reactions were prepared using SYBR® Green Quantitative RT-qPCR Kit (Sigma-Aldrich, St. Louis, MO, USA) and carried out on Applied Biosystems 2720 Thermal Cycler with GAPDH as the endogenous control. Primers of PTCSC3 and GAPDH were designed and synthesized by Sangon (Shanghai, China). PTCSC3 expression levels were normalized to GAPDH using the 2^−ΔΔCt^ method.

### Vectors and cell transfections

PTCSC3 expression vectors were designed and constructed by GenePharma (Shanghai, China). PTCSC3 siRNA and negative control siRNA were designed and constructed by Sangon (Shanghai, China). Cell transfections were conducted in 10^8^ cells per well of 6-well plates with 10 nM vectors or 40 nM siRNAs using Lipofectamine 2000 Reagent (Invitrogen, Carlsbad, CA, USA) following the manufacturer’s instructions. Cells were incubated with transfection mixtures (Lipofectamine 2000 + vector or siRNA) for 6 h and then incubated with fresh media to reduce cyto-activity. Un-transfected cells were control cells and cells transfected with empty vectors or siRNAs were negative controls. Cells were harvested at 24 h after transfection to perform subsequent experiments.

### Cell apoptosis assay

Cell apoptosis assay was performed to investigate the effects of PTCSC3 overexpression and silencing on osteoblast and osteoclast apoptosis. Briefly, cells were harvested, prepared as single-cell suspensions in serum-free media, and adjusted to 3 × 10^4^ cells per ml. Cell suspensions were transferred to a 6-well plate with 2 ml cell suspension in each well and cultured for 36 h. After that, cells were digested with 0.25% trypsin, stained with Annexin V-FITC and propidium iodide (Dojindo, Japan), and subjected to flow cytometry to detect apoptotic cells.

### Statistical analysis

Data of 3 replicate experiments were expressed as the mean ± standard deviation (SD). All statistical analyses were performed using GraphPad Prism 6 (CA, USA) software. Diagnostic potentials of plasma PTCSC3 for osteoporosis were evaluated by performing receiver operating characteristic (ROC) curve analysis with healthy volunteers as the true negative cases and osteoporosis patients as the true positive cases. Comparisons between 2 groups and among multiple groups were performed by unpaired t test and one-way ANOVA plus Tukey test, respectively. The 80 patients were divided into high and low plasma PTCSC3 level groups with the median plasma PTCSC3 level as a cutoff value. Correlations between patients’ clinical data and plasma PTCSC3 expression levels were analyzed using Chi-squared test. *p* < 0.05 was considered statistically significant.

## Results

### PTCSC3 was upregulated in osteoporosis and positively correlated with osteoporosis stages

Plasma PTCSC3 levels in 80 patients with osteoporosis and 80 healthy volunteers were measured by RT-qPCR. Compared with the corresponding controls groups, plasma PTCSC3 levels were significantly increased in each osteoporosis group (Fig. 1, *p* < 0.01). In addition, plasma PTCSC3 levels were obviously increased with clinical stages increasing while were not significantly different among the 4 control groups. Chi-squared test showed that plasma PTCSC3 levels were not significantly correlated with patients’ gender, sedentary lifestyle, alcohol abuse, tobacco smoking, low calcium intake, and family history (Table 2). Therefore, PTCSC3 is likely an independent determinant of osteoporosis. Moreover, RT-PCR was performed to detect PTCSC3 in osteoblast culture medium and fresh medium. As shown in Additional file 1: Fig. S2, PTCSC3 was detected in osteoblast culture medium but not in fresh medium.

**Fig. 1:** Plasma PTCSC3 was upregulated in osteoporosis and positively correlated with osteoporosis stages. RT-qPCR showed that plasma PTCSC3 levels were significantly increased in each osteoporosis group compared with corresponding control groups. In addition, plasma PTCSC3 levels were obviously increased with the clinical stages increasing. By contrast, no significant differences in plasma PTCSC3 levels were found among the 4 control groups. *, *p* < 0.01

**Table 2:** Correlations between patients’ clinical data and the expression of PTCSC3

Items	Groups	Cases	High-expression	Low-expression	χ^2^	*p* value
Gender	Male	40	23	17	1.80	0.18
	Female	40	17	23		
Sedentary lifestyle	Yes	20	12	8	1.07	0.30
	No	60	28	32		
Alcohol abuse	Yes	37	20	17	0.45	0.50
	No	43	20	23		
Tobacco smoking	Yes	44	24	20	0.81	0.37
	No	36	16	20		
Low calcium intake	Yes	19	12	7	1.73	0.19
	No	61	28	33		
Family history	Yes	22	14	8	2.26	0.13
	No	58	26	32		

### Altered plasma PTCSC3 levels separated each stage of osteoporosis from corresponding controls groups

The diagnostic potentials of plasma PTCSC3 for osteoporosis were evaluated by ROC curve analysis with healthy volunteers as the true negative cases and corresponding osteoporosis patient group as the true positive cases. For stage I osteoporosis, the area under the curve (AUC) was 0.92, with a standard error (SE) of 0.039 and a 95% confidence interval (CI) of 0.84–1.00 (Fig. 2A). For stage II osteoporosis, the AUC was 0.90, with a SE of 0.043 and a 95% CI of 0.82–0.99 (Fig. 2B). For stage III osteoporosis, the AUC was 0.99, with a SE of 0.0065 and a 95% CI of 0.98–1.10 (Fig. 2C). For stage IV osteoporosis, the AUC was 0.99, with a SE of 0.0098 and a 95% CI of 0.97–1.10 (Fig. 2D).

**Fig. 2:** Altered plasma PTCSC3 levels separated each stage of osteoporosis from corresponding controls groups. The role of plasma PTCSC3 in the diagnosis of stage I (**A**), II (**B**), III (**C**) and IV (**D**) osteoporosis was analyzed using ROC curve analysis with patients with osteoporosis at each stage as the true positive cases and corresponding controls as the true negative cases

### PTCSC3 positively regulated osteoblast apoptosis

PTCSC3 overexpression and silencing were achieved in osteoblasts at 24 h after transfection (Fig. 3A, *p* < 0.05). Cell apoptosis assay results showed that PTCSC3 overexpression promoted (Fig. 3B, *p* < 0.05) while PTCSC3 silencing inhibited osteoblast apoptosis compared with control (C) and negative control (NC) (Fig. 3C, *p* < 0.05).

**Fig. 3:** PTCSC3 positively regulated osteoblast apoptosis. PTCSC3 overexpression and silencing were reached in osteoblasts at 24 h after transfection (**A**). PTCSC3 overexpression promoted (**B**) while PTCSC3 silencing (**C**) inhibited osteoblast apoptosis. *, *p* < 0.05

### PTCSC3 had no regulatory effect on osteoclast apoptosis

PTCSC3 overexpression and silencing were achieved in osteoclasts at 24 h after transfection (Fig. 4A, *p* < 0.05). Cell apoptosis assay results showed that PTCSC3 overexpression (Fig. 4B) and silencing (Fig. 4C) did not affect osteoclast apoptosis compared with control (C) and negative control (NC).

**Fig. 4:** PTCSC3 had no regulatory effects on osteoclast apoptosis. PTCSC3 overexpression and silencing were reached in osteoclasts at 24 h after transfection (**A**). *, *p* < 0.05. PTCSC3 overexpression (**B**) and silencing (**C**) did not affect osteoclast apoptosis

## Discussion

Osteoporosis is a common clinical bone disease, but its molecular mechanism is unclear. Our study mainly explored the role of PTCSC3 in osteoporosis and found that PTCSC3 is upregulated in osteoporosis and may improve the conditions of osteoporosis.

Early diagnosis of osteoporosis is challenging due to lacking obvious clinical symptoms at stage I and II [15]. Most osteoporosis patients are diagnosed at stage III, in which bones already become too thin to withstand normal stress and bone breaks are common. Recent studies have identified some biomarkers for osteoporosis. However, clinical applications of these biomarkers are limited by either their invasive nature or low diagnostic sensitivity and specificity [16, 17]. In the present study, we identified plasma PTCSC3 upregulation in osteoporosis patients. Furthermore, upregulation of plasma PTCSC3 separates stage I and II osteoporosis patients from the healthy controls. Due to the non-invasive nature of plasma preparation, plasma circulating PTCSC3 may serve as a potential biomarker for the early diagnosis of osteoporosis. However, more clinical trials are needed to further confirm this hypothesis.

Osteoblasts and osteoclasts are key players in the pathogenesis of osteoporosis [18]. Osteoblasts create new bones, while osteoclasts secrete enzymes and acids on bone surface to disintegrate bones [19]. Therefore, decreased osteoblast activity and increased osteoclast activity are common in osteoporosis patients [18], and activating osteoblasts and deactivating osteoclasts are the common targets for treating osteoporosis [20]. In the present study, we found that PTCSC3 positively regulates osteoblast apoptosis but has no effect on osteoclast apoptosis. Therefore, inhibiting PTCSC3 is considered a target for osteoporosis treatment. However, the molecular mechanism underlying the regulatory effects of PTCSC3 on osteoblasts is unknown. It has been reported that PTCSC3 may interact with other molecular factors, such as Wnt/β-catenin, to affect cell apoptosis [21]. More studies, including in vivo animal model investigations, are needed to investigate the involvement of Wnt/β-catenin and other factors in PTCSC3-regulated osteoblast apoptosis.

## Conclusion

PTCSC3 is upregulated in osteoporosis and PTCSC3 downregulation may serve as a target for osteoporosis treatment by inhibiting osteoblast apoptosis.

## Supplementary Information

**Additional file 1.** **Supplemental Figure 1.** Our preliminary deep sequencing analysis revealed altered PTCSC3 expression in osteoporosis. T: osteoporosis groups; ***, *p* < 0.001. **Supplemental Figure 2.** RT-PCR detection of PTCSC3 in medium of osteoblasts and fresh medium.

## Data Availability

The datasets generated during and analyzed during the current study are not publicly available due to further analysis of our data for our future paper, but are available from the corresponding author on reasonable request.

## Abbreviations

lncRNAs: Long non-coding RNAs
RT-qPCR: Real-time quantitative PCR
